# Identifying PIF1 as a Potential Target of Wenxia Changfu Formula in Promoting Lung Cancer Cell Apoptosis: Bioinformatics Analysis and Biological Evidence

**DOI:** 10.1155/2021/9942462

**Published:** 2021-09-24

**Authors:** Xiangjun Yin, Dongfang Kan, Jiazhao Ruan, Delong Wang, Yi Chai, Shengqi Huang, Beiying Zhang, Jixin Wang, Xuming Ji

**Affiliations:** ^1^School of Basic Medical Sciences, Zhejiang Chinese Medical University, Hangzhou 310053, China; ^2^Innovative Institute of Chinese Medicine and Pharmacy, Shandong University of Traditional Chinese Medicine, Jinan 250355, China; ^3^Zhejiang University-University of Edinburgh Institute, Zhejiang University, Hangzhou 310058, China; ^4^Key Laboratory of Neuropharmacology and Translational Medicine of Zhejiang Province, Hangzhou 310053, China; ^5^Academy of Chinese Medical Sciences, Zhejiang Chinese Medical University, Hangzhou 310053, China

## Abstract

Lung cancer remains the leading cause of cancer-related deaths worldwide. Traditional Chinese medicine (TCM) is a valuable resource of active natural products and plays an important role in cancer treatment with the advantages of high efficiency and safety. Wenxia Changfu formula (WCF) is modified from Dahuang Fuzi decoction from Han Dynasty and has been used for treating lung cancer in China. Our previous research showed that WCF had an antitumor effect in vivo and in vitro, while the mechanism has not been well illustrated. In this study, the effect of WCF on the proliferative ability in three lung cancer cells and one noncancerous human cell line was evaluated by 3-(4,5-dimethylthiazol-2-yl)-2,5-diphenyltetrazolium bromide (MTT) assay. WCF suppressed A549, H460, and PC-9 cell viability in a dose-dependent manner, with no inhibition of noncancerous MRC-5 cells after 48 h treatment with WCF (0–50 mg/mL). Furthermore, we screened for genes in A549 cells using four WCF-treated samples and four control samples on a gene expression profile microarray. 21 genes were significantly downregulated by WCF, which may potentially play an important role in the proliferation of A549 cells. High-content screening evaluated whether silencing the 21 genes affected A549 cell growth. The results showed that PIF1 knockdown exhibited the most potent inhibition of cell proliferation compared with the other genes. Downregulation of PIF1 increased A549 cell apoptosis and the activity of caspase 3/7. Besides, RT-PCR showed that the expression levels of PIF1 mRNA decreased significantly in A549, H460, and PC-9 cells after WCF treatment. In conclusion, the present observations indicate that WCF may inhibit lung cancer cell proliferation by promoting apoptosis via regulating the expression of PIF1.

## 1. Introduction

Lung cancer remains one of the most frequently diagnosed cancers and is the leading cause of cancer-related deaths, with >1.7 million deaths worldwide [1, 2]. Among these cases, 80–85% of the total incidence is non-small-cell lung cancer (NSCLC) [3, 4]. Over 60% of lung cancer patients are diagnosed at an advanced stage when the tumor cannot be treated by surgical resection any more, chemotherapy and radiation therapy are still the mainstays of treatment for patients with lung cancer [5, 6]. Despite recent advances in the diagnosis and treatment of lung cancer, the five-year survival rate remains ∼23% [7]. It is still urgent to discover potential therapeutic strategies to improve the prognosis of lung cancer patients [8].

Natural products have played a key role in drug discovery of cancer [9]. It was found that 62 (33.5%) of the total number of small-molecule anticancer drugs approved by FDA in the past 39 years were derived from natural products or their derivatives [10]. Compared with typical synthetic small-molecular libraries, “bioactive” compounds in natural products cover a wider area of chemical space [11]. As a valuable resource of active natural products, traditional Chinese medicine (TCM) plays an important role in lung cancer treatment with unique advantages of high efficiency and minimal side effects [12, 13]. It has an indispensable effect on preventing lung cancer cell proliferation, migration, invasion, enhancing the efficacy, and reducing the side effects of chemotherapy and radiotherapy [14, 15].

Wenxia Changfu formula (WCF) is modified from Dahuang Fuzi decoction which was first recorded in *Synopsis of Golden Chamber* (Jingui Yaolue) written by Zhang Zhongjing from Han Dynasty and is widely used for treating lung cancer in China. It comprises four Chinese herbal ingredients, including *Panax ginseng* C.A. Mey (Araliaceae) (Renshen), *Rheum palmatum* L. (Polygonaceae) (Dahuang), *Aconitum carmichaelii* Debeaux (Ranunculaceae) (Fuzi), and *Angelica sinensis* (Oliv.) Diels (Apiaceae) (Danggui). Previous studies have demonstrated that WCF has a significant antitumor effect as it inhibits the A549 cell line proliferation and induces lung cancer cell apoptosis [16, 17]. Furthermore, WCF effectively enhances chemotherapeutic efficacy and reverses multidrug resistance mediated by cell adhesion in lung cancer cells, the mechanism of which may be related to the integrin *β*1 signaling pathway [18, 19]. Herb formula of TCM is characterized by multitarget, multibiological process and multipathway [20]. However, how WCF exerts antitumor effects via promoting apoptosis has not been well illustrated.

In the present study, the effect of WCF on the proliferation of three lung cancer cells was investigated and then the mechanism was further explored by using microarray analysis, high-content short hairpin RNA (shRNA) screening, etc. Finally, we demonstrate that WCF inhibits lung cancer cell proliferation and promotes apoptosis via decreasing PIF1 expression. The result provides insight into the molecular mechanism of WCF in treating lung cancer and helps us better use WCF clinically.

## 2. Materials and Methods

### 2.1. Preparation of WCF

WCF is composed of *Panax ginseng* C.A. Mey (Araliaceae) (9 g), *Aconitum carmichaelii* Debeaux (Ranunculaceae) (12 g), *Rheum palmatum* L. (Polygonaceae) (12 g), and *Angelica sinensis* (Oliv.) Diels (Apiaceae) (6 g). All crude herbs were purchased from Shandong ZhongLu Hospital (Jinan, China) in June 2018. The authentication was performed by Dr. Feng Li from Shandong University of Traditional Chinese Medicine (Jinan, China). Voucher specimens (No. WCF4-A, B, C, D) were deposited at Affiliated Hospital of Shandong University of Traditional Chinese Medicine (Jinan, China).

The WCF extract was prepared according to the previously reported methods [19]. In brief, the raw herbs *Panax ginseng* and *Aconitum carmichaelii* were decocted for 2 h after they were macerated for 1 h, and then *Angelica sinensis* and *Rheum palmatum* were added and decocted for 0.5 h and 0.25 h, respectively. Finally, the filtrates were concentrated to 1.6 g/mL and stored at −20°C. The concentrations of WCF in this study refer to the crude drug concentrations.

### 2.2. UHPLC/MS Analysis of WCF

The UHPLC/MS analysis was performed according to the procedure we had reported elsewhere [18]. In brief, UHPLC analysis was performed on an UltiMate 3000 RS system (Thermo Fisher Scientific, San Diego, CA). The Thermo Hypersil GOLD column (2.1 mm × 100 mm, 1.9 *µ*m) was applied for all analyses. The mobile phase was composed of A (0.1% formic acid in acetonitrile) and B (0.1% formic acid in water) with a linear gradient elution: 0–5 min, A: 2–20%; 5–10 min, A: 20–50%; 10–25 min, A: 50–95%; 26–30 min, A: 2%. The flow rate of the mobile phase was 0.3 mL/min, and the injection volume was 5 *µ*L. The column temperature was maintained at 35°C.

Mass spectrometry was performed on a *Q* Exactive high-resolution mass spectrometer (Thermo Fisher Scientific, San Diego, CA) and operated using an electrospray source in the positive and negative modes. The operating parameters were as follows: spray voltage, 3.8 kV; capillary temperature, 300°C; sheath gas pressure, 40 arb; aux gas heater temperature, 350°C. Data acquisition and processing were performed using CD 2.1 software (Thermo Fisher), and then they were contrasted with databases (mzCloud, mzVault, and ChemSpider).

### 2.3. Cell Culture and Reagents

Human NSCLC cell lines A549, H460, and PC-9 and human normal fibroblast cell line MRC-5 were purchased from the Chinese Academy of Sciences (Shanghai, China). A549, H460, and PC-9 cells were cultured in RPMI 1640 (Gibco, USA) media supplemented with 10% fetal bovine serum (Sijiqing Bioengineering Material Co., Ltd, China), 100 U/mL penicillin, and 100 *µ*g/mL streptomycin (Gibco, USA) at 37°C in a humidified atmosphere containing 5% CO_2_. MRC-5 cells were maintained in DMEM/F12 media supplemented with 10% fetal bovine serum and 1% penicillin-streptomycin at 5% CO_2_, 37°C.

### 2.4. 3-(4,5-Dimethylthiazol-2-yl)-2,5-diphenyltetrazolium Bromide (MTT) Assay

Cell proliferation was measured using MTT assay. Cell densities of 5 × 10^3^ (A549, MRC-5, and PC-9) or 4 × 10^3^ (H460) cells per 100 *µ*L were seeded into each well in 96-well plates for 12 h; then, they were randomly divided into 5 groups: control group (without WCF) and WCF groups (treated with 100.0, 50.0, 25.0, and 12.5 mg/mL WCF, respectively) and cultured for 48 h at 37°C in 5% CO_2_. Next, 20 *µ*L MTT solution was added to each well. After incubating for 4 h, the medium was removed and the formazan crystals were dissolved by adding 150 *µ*L DMSO. The absorbance was measured using an ELISA reader (SpectraMax M3, Molecular Devices, USA) at a wavelength of 490 nm.

### 2.5. Microarray Analysis and Quantitative Real-Time PCR

Total RNA was extracted with TRIzol reagent (Superfec, China) from lung cancer cell line samples and qualified using a Thremo NanoDrop 2000 (Thermo Fisher Scientific, USA) and an Agilent 2100 Bioanalyzer (Agilent Technologies, USA). Four WCF-treated samples and four negative control samples were used for microarray analysis using the human GeneChip PrimeView array (Affymetrix). Images were captured using a GeneChip Scanner 3000 and analyzed with GeneChip GCOS 1.4 software (Affymetrix). Differentially expressed genes (DEGs) were identified as the expression fold change was >2 and the *P* value was <0.05. For RT-PCR analysis, cDNA synthesis was performed using the M-MLV reverse transcriptase kit (Promega) after total RNA extraction. The real-time PCR was performed in triplicate on a LightCycler 480 System (Roche), and the data were analyzed by using the 2^−△△Ct^ method. GAPDH was used as an internal control.

### 2.6. High-Content Screening and Cell Growth Curve Analysis

The effects of 21 candidate target genes on A549 cell proliferation were detected by high-content screening (HCS). In brief, A549 cells were transfected with shRNA lentivirus targeting candidate target genes or negative control lentivirus after they were seeded at 2000 cells per well in 96-well plates. The GFP expression was observed by using a fluorescence imaging microscope. Cells were collected for further experiments when they reached 80% confluence. Growth of cultured cells was monitored every day for continuous 5 days using the Celigo Image Cytometer (Nexcelom). By adjusting the input parameters of the analysis settings, the number of cells with green fluorescence in each scanning well was calculated. Based on these data, cell proliferation curves were established for target genes or negative control. The cell proliferation ratio of each gene was obtained by comparing the number of cells at each time point with the cell count on day 1, and the cell proliferation curve was produced using the fold change in proliferation. The fold change of each target gene or negative control was calculated as cell count on day 5/cell count on day 1. The gene with a fold change of ≥2 would be identified as a potential target gene which was related to cell proliferation.

### 2.7. Apoptosis Analysis

The Apoptosis Detection Kit (eBioscience) was used for apoptosis analysis according to the manufacturer's instructions. Cells were washed with ice-cold D-Hanks followed by a binding buffer, and then they were resuspended in 1000 *μ*L binding buffer containing 10 *μ*L Annexin V-APC staining solution. The cells were incubated in the dark for 15 min at room temperature, and then the percentage of apoptosis was analyzed by FACS (Millipore). All samples were tested three times.

### 2.8. Caspase 3/7 Activity Analysis

The activity of caspase 3/7 was detected by Caspase-Glo^®^ 3/7 Assay (Promega) according to the kit instruction. Cells were seeded in 96-well plates at 1 × 10^4^ cells per well, and 100 *μ*L Caspase-Glo^®^ 3/7 Reagent was added to each well. The plates were placed on a shaker and shaken at 300–500 rpm for 30 min. Then, the cells were incubated at room temperature for 1-2 h according to the cell conditions. The luminescence was recorded with the GloMax^®^ System.

### 2.9. Statistical Analysis

Data are presented as mean ± SD (standard deviation). Statistical analysis was conducted using SPSS 26.0 (IBM). Statistical differences between two groups were assessed using the independent Student's *t* test, and differences among three or more groups were assessed using one-way ANOVA. A *P* value of <0.05 was considered statistically significant.

## 3. Results

### 3.1. UHPLC/MS Analysis of the Chemical Profile of WCF

UHPLC/MS was applied to analyze and identify the chemical composition of WCF. Through the standard comparison, literature review, and disassociation rules, 15 components were identified. The results are shown in Table 1.

### 3.2. WCF Inhibits Lung Cancer Cell Proliferation

To investigate the effect of WCF on lung cancer cell proliferation, we assessed the cell viability of A549, H460, and PC-9 cells treated with WCF or negative control at 48 h by MTT assay. The results showed that the viability of these three cells decreased in a dose-dependent way when exposed to WCF for 48 h (Figure 1(a)–1(c)). The IC_50_ values were 66.29 mg/mL (A549), 49.53 mg/mL (H460), and 20.46 mg/mL (PC-9), respectively. WCF at a concentration of 50.00 mg/mL (A549 and H460) or 20.00 mg/mL (PC-9) was selected for subsequent experiments. Besides, there was little effect on the viability of MRC-5 cells treated with WCF concentrations ≤50 mg/mL (Figure 1(d)).

### 3.3. Identification of PIF1 as a Potential Target for WCF in Treating Lung Cancer

Microarray experiments comparing 4 pairs of WCF-treated samples and negative control samples revealed 3076 DEGs, 1542 of which in WCF-treated samples were upregulated and 1534 were downregulated (Figure 2(a)). To identify novel oncogenes, we focused on 21 downregulated genes that have not been extensively investigated for potential association with lung cancer, including PIF1, GYG2, and PGM2L1 (Figure 2(b)). All 21 candidate genes were silenced in A549 cells *in vitro*, and the results showed that the silence of PIF1 strongly inhibited cancer cell growth (Figure 2(b) and 2(c)). In addition, PIF1 mRNA expression levels in A549, H460, and PC-9 cells were significantly downregulated after WCF treatment (Figures 2(d)–2(f)), indicating that PIF1 may serve as a potential target for WCF in the regulation of lung cancer cells.

### 3.4. PIF1 Promotes Lung Cancer Cell Proliferation *In Vitro*

To further determine PIF1 function in lung cancer cell proliferation, stable PIF1 knockdown in the A549 cell line was established with a lentiviral delivery system, and we confirmed downregulation of both PIF1 protein and mRNA in this cell line (Figure 3(a), 3(b)). PIF1 knockdown suppressed A549 cell proliferation, as measured by Celigo and cell growth curve analysis using a fluorescence imaging system (Figure 3(c)).

### 3.5. PIF1 Knockdown Inhibits Lung Cancer Apoptosis

To explore whether PIF1 promotes lung cancer cell proliferation through regulating cell apoptosis, Annexin V-APC staining was performed by using a flow cytometer. PIF1 knockdown increased the percentage of A549 cells undergoing apoptosis (Figure 4(a), 4(b)), and the activity of caspase 3/7 was increased in the shPIF1 group (Figure 4(c)). These results indicate that PIF1 silencing can inhibit A549 cell proliferation via promoting apoptosis.

## 4. Discussion

In this study, we determined that WCF could significantly inhibit lung cancer cell proliferation and PIF1 was significantly downregulated after WCF treatment. PIF1 knockdown suppressed cell proliferation and promoted cell apoptosis of A549 cells. These results suggest that PIF1 may play a critical oncogenic role in tumor growth and serve as an attractive therapeutic target after WCF treatment in lung cancer.

TCM is an important part of complementary and alternative medicine and has been increasingly used in the past few decades, which affects the overall survival of lung cancer patients [21]. According to TCM theory, Yang deficiency or Qi deficiency, blood stasis, and stagnation are important pathogenic factors for lung cancer, and WCF can warm Yang, strengthen Qi, resolve blood stasis, and eliminate stagnation [19, 22, 23]. Our previous study showed that combination of WCF with cisplatin could significantly inhibit the A549 cell line proliferation *in vitro* and reduce the tumor volume *in vivo*, compared with the cisplatin group, and the apoptosis body was found in tumor cells in the WCF-treated group [16, 17, 19]. WCF has an inhibitory effect on lung cancer cell growth by inducing apoptosis, while the mechanism is still unclear.

Nowadays, microarray bioinformatics has been widely used to identify differentially expressed genes and functional pathways that participate in lung cancer development [24]. There are thousands of genes within the human body, and the expression of these genes varies from tissue to tissue depending on the cell type; thus, the traditional gene-by-gene method is not powerful enough to define gene changes at the genome level in a single experiment [25]. Therefore, in this study, we used microarray technology to screen the differentially expressed genes between the control A549 cells and the WCF-treated A549 cells to identify the potential targets of WCF in inhibiting lung cancer cell proliferation. Finally, 21 oncogenes were identified, and we selected PIF1 to further confirm its biological function in A549 cells based on the high-content screening results. PIF1 is a multifunctional helicase and plays important roles in mitochondrial and nuclear genome maintenance, telomere length regulation, unwinding of G-quadruplex structures, and DNA synthesis during break-induced replication [26–28]. It is conserved in most eukaryotes and some prokaryotes [29, 30]. The human genome encodes a single PIF1 gene; splice variant of human PIF1 (hPIF1) localizes to both the nucleus and mitochondria [31, 32].

At present, the cellular functions of hPIF1 are still unclear. A few studies have reported that PIF1 was essential for human tumor cell proliferation, including HCT116 cells, HeLa cells, and HEY cells [33–35]. hPIF1 played an important role in DNA replication, especially under oncogenic stress [31]. It had been reported that PIF1 depletion could reduce the survival of neuroblastoma cells by triggering apoptosis, which was dependent on the activity of caspase-3, while nonmalignant cells were not affected by PIF1 depletion [36]. hPIF1 has therefore been proposed as a cancer therapy target [28]. The mechanism may be related to its effect on maintaining mitochondrial stability in response to reactive oxygen species (ROS) [37]. ROS are essential for the initiation, progression, and metastasis of cancer, and altered ROS levels in cancer cells are one of the reasons for recurrence/relapse [38]. By increasing ROS production, cancer cells and drug resistance can be eliminated, which has been demonstrated by a large number of FDA-approved anticancer drugs [38, 39], while PIF1 is involved in reducing the mitochondrial DNA damage caused by ROS [40]. Currently, the role of PIF1 in lung cancer cells is still not reported. In this research, we found that PIF1 played an important role in promoting lung cancer cell proliferation, and it might be a critical target for WCF. However, further studies using appropriate animal models are still needed to confirm the potential of PIF1 as an anticancer drug target.

## 5. Conclusions

We found that WCF inhibited the proliferation of NSCLC cells and downregulated the expression of PIF1 and stable PIF1 knockdown suppressed A549 cell growth and promoted apoptosis. In summary, PIF1 may be a critical gene that regulates lung cancer cell proliferation and apoptosis, which may serve as a potential target of WCF in treating lung cancer.

## Figures and Tables

**Figure 1:** WCF treatment resulted in dose-dependent inhibition of proliferation in NSCLC cell lines. (a) Viability of A549 cells after WCF treatment. (b) Viability of H460 cells after WCF treatment. (c) Viability of PC-9 cells after WCF treatment. (d) Viability of MRC-5 cells after WCF treatment.  ^*∗*^ ^*∗*^*P* ˂ 0.01.

**Figure 2:** Microarray analysis, quantitative real-time PCR, and high-content screening identified PIF1 as a potential target for WCF in inhibiting lung cancer cell proliferation. (a) Heat map which was used to compare gene expression profiles in A549 cells. (b) Representative fluorescence images of high-content screening for PIF1, GYG2, and PGM2L1 on the growth of A549 cells. (c) A total of 21 genes were selected for validation by high-content screening, and data were presented as fold change and normalized to cell number on day 1. (d) PIF1 mRNA expression in A549 cells treated with WCF or negative control. (e) PIF1 mRNA expression in H460 cells treated with WCF or negative control. (f) PIF1 mRNA expression in PC-9 cells treated with WCF or negative control.  ^*∗*^ ^*∗*^*P* ˂ 0.01.

**Figure 3:** PIF1 promotes A549 cell proliferation *in vitro*. (a) Representative fluorescence images of A549 cells transfected with shPIF1 or shCtrl for 72 hours. (b) PIF1 mRNA expression in A549 cells transfected with shPIF1 or shCtrl for 72 hours. (c) Cell growth curve analysis comparing PIF1 knockdown (shPIF1) with negative control (shCtrl) A549 cells.  ^*∗*^ ^*∗*^*P* ˂ 0.01.

**Figure 4:** PIF1 regulates A549 cell proliferation via promoting apoptosis. (a, b) Cell apoptosis was analyzed using Annexin V-APC staining, followed by a flow cytometer. (c) Activity of caspase 3/7 was determined in A549 cells transfected with shPIF1 or shCtrl.  ^*∗*^ ^*∗*^*P* ˂ 0.01.

**Table 1:** Identification of some chemical constituents in WCF.

No.	Name	Formula	RT (min)	mzCloud best match
1	DL-arginine	C_6_H_14_N_4_O_2_	1.279	93.3
2	L-histidine	C_6_H_9_N_3_O_2_	1.296	91.4
3	Trigonelline	C_7_H_7_NO_2_	1.398	94.6
4	Proline	C_5_H_9_NO_2_	1.476	85.1
5	Pyridoxine	C_8_H_11_NO_3_	2.849	86.5
6	N6-methyladenine	C_6_H_7_N_5_	4.161	79.4
7	Indole-3-acetic acid	C_10_H_9_NO_2_	5.915	88.1
8	Neochlorogenic acid	C_16_H_18_O_9_	7.099	82.1
9	*N*-acetyl-L-phenylalanine	C_11_H_13_NO_3_	9.022	76.2
10	Glycitein	C_16_H_12_O_5_	13.195	83
11	Betulin	C_30_H_50_O_2_	14.324	80.2
12	Genistein	C_15_H_10_O_5_	15.435	82.2
13	*α*-eleostearic acid	C_18_H_30_O_2_	16.855	93
14	Oleamide	C_18_H_35_NO	17.057	92.3
15	Rubiadin	C_15_H_10_O_4_	17.161	89.6

## Data Availability

The data that support the findings of this study are available from the corresponding author on reasonable request.
